This article has been retracted.

# Design and Application of Legally Valid Payment Templates Based on Linking Contracts

**DOI:** 10.1155/2022/1331237

**Published:** 2022-07-18

**Authors:** Yue Zhu

**Affiliations:** School of Law, Tsinghua University, Beijing 100084, China

## Abstract

Smart contracts are widely employed in many industries as a result of the high-quality development of science and economic technology, as well as the introduction of blockchain, which can automatically conduct retrieval, verification, and payment tasks. Smart contracts as an emerging topic, particularly the study of smart legal contracts, must remain forward-looking, and the smart contract sector cannot wait for the legal status of smart contracts to be resolved before advancing. The relative lag of the law becomes unavoidable due to the unassembled and unpredictable character of the law and thus its legislation. In this paper, we explore the incorporation of smart contracts into the scope of legal regulation, the construction of a series of systems for smart contracts, and the prognosis of smart contracts in terms of contract logic, arbitration process, and formal verification from the current law. Furthermore, a smart contract payment template based on semantic-aware graph neural networks is proposed to address the traditional smart contract vulnerability detection payment template method's low detection accuracy and high false alarm rate, as well as the neural network-based method's insufficient mining of bytecode-level smart contract features. Experiments comparing the method described in this research to comparable methods reveal that the strategy proposed in this study improves all types of indicators significantly.

## 1. Introduction

With the use and development of smart contracts, the form of smart contract clauses has become more complex and diverse, one of which is the smart contract payment linkage clause, which can connect numerous smart contracts and form various contractual interactive systems. Smart contracts, as a form of transaction, should still essentially belong to the category of contract law regulation. However, due to the characteristics of smart contracts, such as automatic execution, decentralized supervision and irrevocability, and the complexity and diversity of smart contract payment linkage clauses, smart contract payment linkage clauses bring great challenges to the regulation of contract law in terms of validity determination, post facto remedy, and prior regulation [1–3]. The question of how contract law should respond and regulate this is the subject of this paper.

The concept of a smart contract was first proposed by cryptographer Nick Szabo and is defined as “a set of digitally defined promises, including an agreement on which the contracting parties can execute those promises.” Sabo's working theory of smart contracts was not possible because computer programs could not actually trigger payments until the advent of blockchain technology, which allows smart contracts to enable real-world value exchange. The search popularity of linking contracts in Google is shown in Figure 1, which shows a sharp increase in recent years, indicating that this is a meaningful research direction [4–7]. Autonomy, self-sufficiency, and decentralization are three properties of blockchain-based smart contracts. Self-sufficiency indicates that the smart contract can generate its own revenue by offering services; autonomy means that the contract runs automatically once it is installed; decentralization means that it does not rely on a centralized server and runs automatically through network nodes [5].

International legal research on blockchain smart contracts has gone further than that in China, and there are preliminary explorations of the legal aspects of smart contracts [8, 9]. These investigations focus on the legal properties of smart contracts and the relationship between smart contracts and existing contract law. As far as the legal attributes of smart contracts are concerned, there is a great deal of controversy among international scholars, mainly including the following views: self-help behavior. This view is that the self-execution feature of smart contracts indicates that they are an ex-ante self-help act, because they can be executed without judicial force. Max Reskin, J.D., of New York University, is a proponent of this view, citing the example of a smart car ignition device that prevents the car from being started if the owner fails to pay the bank loan on time, which was agreed upon at the time of the contract between the owner and the bank and the seller of the car. Apparently, the smart contract functions similarly to the car ignition. Escrow agent argument [10]: this view is that instead of calling it a smart contract, it should be called a “smart agent.” In a normal escrow agent arrangement, the parties to a transaction place the subject matter of the contract in the custody of a third party, who is entrusted with executing the contract once the parties have reached an agreement, because they do not trust each other. A smart contract acts as such a third party, with the parties placing blockchain assets in a contract that is automatically executed once the contract conditions are met. According to Nicolas Cornell, a smart contract is still a contract in the sense of contract law. According to the Restatement Second of the United States Law of Contracts, a contract is a promise or series of promises for which the law will provide relief in the event of a breach or which the law treats as an obligation enforceable by law. The self-executing function of a smart contract does not require legal compulsion, but it does not mean that a smart contract cannot be legally compelled either [11–13]. Therefore, in the opinion of these two professors, as long as a smart contract can change the rights and obligations between the parties according to their intention, it still belongs to a contract in the sense of contract law [14].

Although existing smart contract methods address the issue of low automation in traditional methods, they still have the following flaws: no semantic elements of smart contract bytecode are extracted, and the detection effect is poor. The graph neural network-based smart contract vulnerability detection payment template method focuses on the graph structure and ignores feature extraction of smart contract bytecode semantic features, instead focusing on the neural network's learning of function invocation relationships, which results in the loss of a significant amount of semantic information in the nodes and makes it difficult to generate high-quality node representations (high-quality node representations can be used to measure node similarity and are also a prerequisite for accurate node classification). Some methods have less coverage on payment template types and are not well adapted for emerging vulnerabilities. In order to solve the above problems of smart contract vulnerability detection payment template methods, this paper proposes a semantic-aware graph neural network-based smart contract payment template method (L-GCN) for smart contracts in the actual deployment environment to solve the problem of low accuracy of vulnerability detection payment template methods with high false alarm rate and difficulty in covering complex smart contract function call relationships. The main advantages of the method are proposing a semantic extraction method based on smart contract bytecodes, applying the natural language processing method to the semantic extraction of smart contract bytecode instructions, using semantic vectors instead of low-dimensional vectors, and generating a higher quality node representation; using GCN's high performance in processing non-Euclidean structure samples, merging semantic information for vulnerability detection payment templates, and improving node feature learning; the importance of semantic features for smart contract vulnerability detection payment templates is illustrated by experimental design.

The paper's organization paragraph is as follows. The related work is presented in Section 2.  Section 3 analyzes the methodology of the proposed work.  Section 4 discusses the experiments and results. Finally, in Section 5, the research work is concluded.

## 2. Related Work

### 2.1. Third-Party Payment Encryption Scheme

A ciphertext search system relying on a third party usually includes three subjects: the data owner, the user, and the cloud server, as shown in Figure 2. In the cloud server (third-party)-based ciphertext search scheme, the data owner encrypts the file using searchable encryption algorithm and at the same time extracts the keywords encrypted in the file and builds a secure index table and sends the file ciphertext and index together to the cloud server [15–17]. When a user needs to access a file containing a certain keyword, he sends the search credentials of the obtained keyword to the cloud server, which matches the search credentials with each file and finally returns the successfully matched file to the user. The user decrypts the ciphertext to obtain the desired file [18]. The server is honest and curious in the whole process, and the user needs to pay the service fee to the server before retrieving, and the server performs the search task honestly and returns the search results to the user. However, the search results returned by the server may be incorrect or may not be returned as required, and then, it is necessary for the authority to judge and arbitrate, even if the user is refunded the fee paid, but the whole process is complicated and long, which is unfair to the user, and this is the shortcoming of traditional ciphertext search based on third-party cloud servers [19]. This is also the drawback of traditional third-party cloud-based cipher search.

### 2.2. Linking Contract-Based Payment Scheme

Smart contracts can automatically perform retrieval, verification, and payment functions. In this paper, we use smart contracts to solve the verification and fair payment problems in traditional ciphertext search. The smart contract-based ciphertext search and fair payment scheme contains five roles: data owner, server, user, and smart contract [20, 21]. As shown in Figure 3, the data owner can predefine the access policy in the ciphertext, and only when the user's attribute set satisfies the access policy can the decryption key be retrieved, resulting in the original ciphertext of the ciphertext validated by the smart contract search. Smart contracts have the ability to read and write stored files, send messages to users or servers, and deposit funds into the contract account on a temporary basis, temporarily deposit service fees in the contract account, temporarily deposit inquiry fees in the contract account, and smart contracts can verify the search results [22–23].

### 2.3. The Legal Properties of Smart Contract Payments

Smart contract payment linkage clause is not a concept in contract law, but refers to the contract clause that uses other smart contracts as the execution trigger, which can link the effectiveness and execution of multiple smart contracts. According to some scholars, smart contracts can be used to link many contracts into various kinds of contractual interactive network systems, which are called “linking contracts,” and the smart contract payment linkage clause acts as such a linking node. Ethernet is the most widely used smart contract platform, and as an open-source platform, it can use the Turing-complete language, allowing users to write a variety of smart contract terms according to their needs. While the linguistic logic of the contract code makes smart contract payment linkage clauses seem similar to conditional contracts in contract law, in fact their application goes far beyond the meaning of conditional contracts. In the various contractual interactive systems formed by Ethernet, similarities can be found with many types of contracts governed by existing contract law, which may exist in the form of contract linkage, contract conjunctions, and other similar forms, in addition to being similar to contracts with conditional effect. A contract with conditional effect means that the parties agree on the corresponding conditions in the contract, and the occurrence or extinction of the contract effect is determined by the fulfillment or otherwise of the conditions.

The conditions attached to the contract here can be either a legal event or a legal act, so based on the definition of smart contract payment linkage clause in this paper, it seems to be concluded that all smart contract clauses with uncertain future contractual transaction behavior as a precondition are smart contract payment linkage clauses. However, in fact, many smart contracts are usually unilateral contracts deployed unilaterally by the user on the blockchain, and multiple smart contracts linked together may also express the same contractual relationship. For example, A and B agree to buy and sell, so A deploys smart contract A on the blockchain, agreeing that “if B pays the corresponding digital currency to this account, then the house corresponding to the digital asset under this account will be transferred to B,” and then, B writes smart contract B to confirm the payment of the corresponding digital currency to A. In this example, smart contract A is executed by smart contract B. Although it is in line with the characteristics of a contract with conditional effect, it is not a smart contract payment linkage clause, because the relationship between the two contracts is a sale and purchase contract according to the transaction purpose of the parties, and the condition predetermined by contract A is not a condition of a contract with conditional effect, but refers to the obligations under the sale and purchase contract. Therefore, the smart contract payment linkage clause in the form of a conditional contract must be manifested by the existence of two or more contractual relationships, and the precondition is a contractual act of uncertainty in the future.

## 3. Methodology

### 3.1. Model Structure

The method proposed in this paper is based on smart contract bytecode implementation. Because most smart contracts on Ethernet are written in bytecode, the method of collecting semantic information from bytecode and merging payment templates from graph neural networks is more suited to the smart contract operating environment. The overall framework of the method is shown in Figure 4.

The overall architecture of the method in this paper consists of four phases:

1. Smart contract bytecode generation phase: based on the smart contract source code in the public dataset, compiled according to the compiler version declared within the contract code to generate bytecode
2. Graph node feature generation phase: dividing nodes from the bytecode to generate CFG and inputting them into GCN for training to generate node features
3. Semantic feature generation phase: the word vector generated by extracting semantic information from the bytecode instructions within each node is input into the LSTM network for training to generate semantic features
4. Obtaining result stage: the vector representation of node features and semantic features are spliced and input into the fully connected layer, mapped to the sample tag space, and the final prediction results are obtained. The 4 parts are described in detail below

### 3.2. Smart Contract Bytecode Generation

Smart contracts run as bytecode when deployed on Ethernet, so it is more practical to generate smart contract bytecode as the basis for vulnerability detection. However, the current public datasets of smart contracts are released in the form of source code, so the datasets need to be compiled to generate bytecode. Smart contract compiler versions are quite sophisticated, and different compiler versions are incompatible with one another, as well as the compiled bytecode. In this paper, we strictly follow the compiler version declared in the source code of each smart contract in the process of compilation to prevent the interference of the detection effect caused by the different bytecodes generated by different compiler versions.

### 3.3. Graph Node Feature Extraction

CFG contains smart contract structure information, which can represent the invocation relationship between functions. In this paper, the nodes are redivided based on smart contract bytecode instructions, which can make the function invocation relationships clearer and enable GCN to better learn control features from CFG. Programs can be converted into symbolic graph representations, and symbolic graph representations are able to preserve the semantic relationships between program elements. The value of various functions differs in the process of identifying smart contract vulnerabilities. This study uses function call relationships to redivide the nodes and builds CFGs from smart contract source code. Each smart contract generated CFG is represented by the nodes in the contract and the edges between the nodes, and the following describes how to obtain the nodes and edges, respectively. After compiling the source code in the dataset to generate bytecode, the bytecode is disassembled to generate bytecode instructions. After determining the function entry, only the end instruction of the function needs to be found to divide a basic block according to the function. A summary of the instructions that represent the end of the basic block is shown in Table 1. Each node represents a basic block, and each basic block does not necessarily cover a complete function, because there are also instruction jumps within the function. A set is used to represent all the nodes in the CFG. After obtaining the nodes, the call relationship between nodes is considered as an edge, representing that the previous function may call the next function. Each node may call multiple nodes and may be called by multiple nodes. Use the set to represent the edges in *E* CFG. gg = (*V*; *E*). After node division and edge construction, use *G* to represent the CFG. The CFG is fed into the GCN for training to obtain the features of the graph. For each layer of the neural network, it can be represented by the following nonlinear function.

(1) $$\begin{array}{c} H^{\left(l+1\right)}=f\left(H^{\left(l\right)},A\right), \end{array}$$

where *l* denotes the number of network layers, *H* input layer and output layer, and *f* is the differentiable function of the neural network; **A** is the adjacency matrix. The classification of the graph by GCN utilizes the feature information of the nodes themselves and the structure information of the graph, and the learning strategy is as follows.

(2) $$\begin{array}{c} \begin{array}{c} \Gamma =\Gamma_{0}+\lambda \Gamma_{\text{reg}},\\ \Gamma_{\text{reg}}=f{\left(X\right)}^{\text{T}}\Delta f\left(X\right), \end{array} \end{array}$$

where Γ_0_ is the supervisory loss of the labeled nodes in the graph, Γ_reg_ is the loss introduced by the graph structure information, *λ* is the weight coefficient, and **X** is the node feature vector matrix, with Δ which represents the Laplace operator of the graph. The hierarchical propagation rule of the GCN model is as follows.

(3) $$\begin{array}{c} f\left(H^{\left(l+1\right)},A\right)=\sigma \left({\tilde{D}}^{-1/2}\tilde{A}{\tilde{D}}^{-1/2}H^{\left(l\right)}W^{\left(l\right)}\right), \end{array}$$

where $\tilde{A}=A+I$, *I* is the unit matrix, **A** is the adjacency matrix added to the self-loop for aggregating the node's own information with all neighboring nodes, **D** is the degree matrix of the **A** matrix, and *σ* denotes the nonlinear activation such as linear rectification function functions.

### 3.4. Node Semantic Information Extraction

The CFG graph that is constructed contains graph structure information. The fundamental blocks of a smart contract are the nodes of the CFG graph, and each basic block consists of a set of instructions from which features must be extracted. Low-latency embedding based on manually selected features leads to a large amount of semantic information loss. Extracting these instructions as node features using natural language processing (NLP) models can maximize the preservation of semantic information. After obtaining the bytecode instructions of each node through node segmentation and bytecode disassembly, the bytecode instructions are treated as natural language processing. First, the instructions are divided into words according to the instructions; then, the sequences are mapped into vector representations, i.e., the subscripts of words in the word set are used as word representations; finally, the instruction vector sequences are input into the LSTM network for training to obtain semantic representations, as show in Figure 5. Considering the temporal order and coherence between instruction information, using LSTM network can solve the gradient disappearance problem, learn the long-distance dependency between instructions, make the sequential nature between instructions fully reflected in the sequence, and preserve the semantic features to the maximum extent. LSTM uses gating mechanism, which consists of input gate, forgetting gate, and output gate as a module, formed by multiple modules with the same structure in series; when the instruction sequence sequentially passes through the LSTM network, the gate structures in these modules will be adjusted to the features that need to be remembered and forgotten, thus obtaining the final generated semantic features with long-range dependencies. The specific formula of the gating mechanism is as follows.

(4) $$\begin{array}{c} \begin{array}{c} f_{t}=\sigma \left(W_{f}x_{t}+U_{f}h_{t-1}+b_{f}\right),\\ i_{t}=\sigma \left(W_{i}x_{t}+U_{i}h_{t-1}+b_{i}\right),\\ o_{t}=\sigma \left(W_{o}x_{t}+U_{o}h_{t-1}+b_{o}\right),\\ c=\tan h\left(W_{c}x_{t}+U_{c}h_{t-1}+b_{c}\right),\\ c_{t}=f_{t}\circ c_{t-1}+i_{t}\circ c,\\ h_{t}=o_{t}\circ \tan h\left(c_{t}\right), \end{array} \end{array}$$

where **x**_*t*_ and **h** are the input and output vectors, respectively; *σ* denotes the sigmoid function; *t* is the time step value; *W* is the weight of the input; *U* is the weight of the cyclic output; **h**_*t*_ is the output gate vector that controls what information the current internal state needs to output to the external state.

### 3.5. Combining Features to Obtain Prediction Results

After obtaining the node features and semantic information features, the two features are stitched together and input to the fully connected layer to combine the two features and map them to the sample labeling space. In order to reduce the isomorphism bias in the classification model, the output of the fully connected layer is obtained and input to the SoftMax layer for normalization.

(5) $$\begin{array}{c} \text{SoftMax}\left(g_{i}\right)=\frac{\exp\left(g_{i}\right)}{\sum_{z=1}^{Z}\;\exp\left(g_{n}\right)}, \end{array}$$

where *g*_*i*_ is the output value of the *i*-th node; *g*_*n*_is the number of output nodes; *z* by SoftMax function can transform the output into a probability distribution to accomplish the goal of prediction. Detection of no vulnerability for positive class samples, with vulnerability for negative class samples, by comparing with the label will have four cases, the four metrics are expressed as

(6) $$\begin{array}{c} \begin{array}{c} F_{\text{acc}}=\frac{\left(n_{\text{TP}}+n_{\text{TN}}\right)}{\left(n_{\text{TP}}+n_{\text{FN}}+n_{\text{FP}}+n_{\text{FN}}\right)},\\ F_{\text{pre}}=\frac{n_{\text{TP}}}{\left(n_{\text{TP}}+n_{\text{FP}}\right)},\\ F_{\text{rec}}=\frac{n_{\text{TP}}}{\left(n_{\text{TP}}+n_{\text{FN}}\right)},\\ F_{1}=2\cdot F_{\text{pre}}\cdot \frac{F_{\text{rec}}}{\left(F_{\text{pre}}+F_{\text{rec}}\right)}, \end{array} \end{array}$$

where *F*_acc_ is defined as accuracy, *F*_pre_ is precision, *F*_rec_ is recall, and *F*_1_ is the *F*1 score.

## 4. Experiments and Results

In this section we define the dataset, experimental setup, and experimental results and analysis in detail.

### 4.1. Dataset

The SmartWild dataset was collected from real-world smart contracts with transactions that were repetitively screened for potentially vulnerable smart contracts, using real Ethereum contract addresses as the unique identifier. Because there are so many different versions of smart contract compilers and they are not all compatible, the bytecode output from source code compilation varies a lot, which can affect the experimental results. Many smart contracts written with older compiler versions are rarely used on Ether. This study leverages the dataset to better imitate the current smart contract situation by filtering out some smart contracts with too early compiler versions and bytecode repeated filtering for the remainder, ultimately using 21437 of them for tests. The SBcurated dataset consists of a part of real-world contracts with vulnerabilities and a part of hand-constructed contracts with vulnerabilities. Contracts: the smart contracts in this dataset are manually tagged with the location and class of vulnerabilities and can be used to evaluate the effectiveness of smart contract analysis tools in identifying vulnerabilities. The dataset has 136 samples. In this paper, we use the above two datasets for vulnerability detection in the experimental part and design comparative experiments to demonstrate the effective enhancement of semantic information for smart contract vulnerability detection and the ability to detect real-world smart contracts with vulnerabilities.

### 4.2. Experimental Setup

First, because the combination of Mythril and Slither provides both accuracy and efficiency, it was chosen to generate labels for the 21437 smart contracts in the SmartWild dataset. The number of training sets is 19437, and the number of testing sets is 2000 in this dataset, which is utilized for both training and testing. These smart contracts are detected using this paper's method (LGCN), compared to Oyente, Smartcheck, and Manticore, three traditional detection tools, and a vulnerability detection method that uses only GCN networks without semantic features (referred to as GCN) for comparison. The evaluation metrics used are accuracy (accuracy), precision (precision), recall (recall), and *F*1 score (*F*1). The ability of this paper's method (L-GCN) to uncover real smart contract vulnerabilities versus classic Oyente, Smartcheck, Manticore, and GCN detection methods is then tested using 136 manually classified smart contracts from the SBcurated dataset. Since all contracts in this dataset are vulnerable, only the accuracy is compared.

### 4.3. Experimental Results and Analysis

The experimental results of the SmartWild dataset are analyzed, and Table 2 shows the results of the performance metrics of smart contract vulnerability detection using five methods on the SmartWild dataset of 21437 real smart contracts.

The experimental data in Table 2 reveals that the L-GCN suggested in this paper outperforms the other four approaches in all four metrics when compared to the other five methods. Among the 4 metrics, the L-GCN method has a large improvement in accuracy, precision, and *F*1 score, but the difference in recall rate among the 5 methods is not large, indicating that all 5 methods focus more on the detection rate for smart contracts with vulnerabilities, while the lower precision metric indicates that the first 4 methods have a high false alarm rate along with a high detection rate, while the LGCN method has the highest recall rate value while improves the precision value, indicating that the method can effectively reduce the false alarm rate. Compared with the GCN method, all four metrics of the L-GCN method increased, indicating that adding semantic information can indeed improve vulnerability detection. It is worth mentioning that the Oyente method has a very high recall value, almost the same as the L-GCN method. The SmartWild dataset is tagged using a combination of smart contract vulnerability detection methods based on symbolic execution, which has some enhancement for the Oyente approach, which is also based on symbolic execution, according to the theory. This experimental result shows that adding semantic features can effectively improve smart contract vulnerability detection, and the smart contract vulnerability detection method proposed in this paper on semantic-aware graph neural network can achieve the goal of improving detection accuracy while reducing the false alarm rate.

Analysis of experimental results for the SBcurated dataset: Table 3 shows the accuracy of vulnerability detection and the number of smart contracts with vulnerabilities detected for 136 smart contracts in the SBcurated dataset using five methods.

The SBcurated dataset contains less data than the SmartWild dataset, but the smart contracts in it are manually categorized and labelled with greater precision, demonstrating the usefulness of the detection methods. The remaining four methods were used to detect all of the samples. From the metrics in Table 3, the detection accuracy and the number of vulnerabilities contained in the semantic-aware smart contract vulnerability detection method (L-GCN) proposed in this paper are higher than those of the other four methods, but the improvement is not as obvious as that of the SmartWild dataset. It is speculated that the possible reason is that the samples in the SmartWild dataset all have vulnerabilities and are therefore all positive class samples, at which point the accuracy is effectively equivalent to the recall rate metric in Table 2. Comparing the recall metric in Table 2 with the accuracy in Table 3 also reveals that the five detection methods rank almost identically on these two metrics. This means that all five approaches have a high detection rate for susceptible contracts, and the detection impact improves as the number of vulnerable contracts in the sample grows larger; however, the L-GCN method suggested in this research still outperforms the other four ways. By counting the contracts with vulnerabilities detected, among all the contracts with vulnerabilities detected by the L-GCN method, there are four contracts with vulnerabilities that are not detected by the first four methods. This experiment shows that when detecting real smart contract vulnerabilities, the semantic-aware graph neural network-based smart contract vulnerability detection method proposed in this paper is more effective and can detect the contracts with vulnerabilities that other methods in the experiment failed to detect.

## 5. Conclusion

In this paper, we propose a fully automated smart contract vulnerability analysis method based on semantic-aware graph neural networks. Due to the unassembled and unpredictable nature of the law and therefore its legislation, the relative lag of the law becomes unavoidable. We combine the good processing ability of neural networks for graph structure with the extraction of semantic information by natural language processing methods and use both function call relationships and learning nodes' own bytecode features in the process of using payment templates and investigate the possibility of adding semantic information to neural networks for smart contracts, in comparison to existing methods. The possibility of adding semantic information to neural networks for intelligent contract vulnerability detection is explored. After extensive experiments, it is shown that the semantic-aware graph neural network-based smart contract vulnerability detection method can effectively improve the detection accuracy and reduce the false alarm rate and has the ability to detect vulnerabilities in real smart contracts.

## Figures and Tables

**Figure 1:** Linking contracts in Google search heat.

**Figure 2:** Cloud server-based ciphertext search solution.

**Figure 3:** Framework diagram of smart contract-based ciphertext search and fair payment scheme.

**Figure 4:** Model architecture.

**Figure 5:** LSTM structure.

**Table 1:** Instructions representing the end of the basic block.

Command	Role
STOP	Stop
SELFDESTRUCT	Self-destruct
RETURN	Return
REVERT	Judgment
INVALID	Invalid
SUICIDE	Delete
JUMP	Jump
JUMPI	Jump

**Table 2:** Performance comparison based on the SmartWild dataset.

Detection method	Accuracy (%)	Precision (%)	Recall rate (%)	*F*1 (%)
Manticore	36.57	31.90	86.32	46.58
Oyente	37.36	33.13	92.73	48.82
Smartcheck	39.72	32.53	81.01	31.09
GCN	68.05	67.42	88.73	76.62
L-GCN	81.40	79.23	92.79	85.48

**Table 3:** SBcurated dataset accuracy.

Detection method	Accuracy (%)	Number of smart contracts containing vulnerabilities
Manticore	79.17	108
Oyente	80.88	110
Smartcheck	71.37	97
GCN	87.50	119
L-GCN	92.65	126

## Data Availability

The datasets used during the current study are available from the corresponding author on reasonable request.
